The article "The Effects of Intensive Blood Pressure Control on Cardiovascular Outcomes Based on 10-Year ASCVD Risk Score: An Analysis of a Clinical Trial" was published in 2021. Journal: Cardiol Res Pract.

# The Effects of Intensive Blood Pressure Control on Cardiovascular Outcomes Based on 10-Year ASCVD Risk Score: An Analysis of a Clinical Trial

**DOI:** 10.1155/2021/6635345

**Published:** 2021-05-11

**Authors:** Alireza Alborzi, Armin Attar, Mehrab Sayadi, Fatemeh Nouri

**Affiliations:** ^1^Department of Cardiovascular Medicine, Shiraz University of Medical Sciences, Shiraz, Iran; ^2^Student's Research Committee, Shiraz University of Medical Sciences, Shiraz, Iran

## Abstract

There is still controversy about whether clinicians should include cardiovascular disease (CVD) risk stratification into the consideration for treatment of hypertension. This was a post hoc analysis of the Systolic Blood Pressure Intervention Trial (SPRINT). A total of 9361 nondiabetic patients without a history of stroke were randomly assigned to the intensive-treatment group (with an SBP target of <120 mm Hg) and the standard-treatment group (with an SBP target of <140 mm Hg). The patients were categorized into four groups based on the Atherosclerotic Cardiovascular Disease (ASCVD) risk score. The groups contained participants with ASCVD < 7.5%, 7.5% ≤ ASCVD <10%, 10% ≤ ASCVD < 15%, and ASCVD ≥ 15%. The incidence of the primary outcome, secondary outcome, and serious adverse events was compared between the two groups. The primary outcome was a composite of nonfatal myocardial infarction (MI), acute coronary syndrome (ACS) not resulting in MI, stroke, acute decompensated heart failure (HF), or death from cardiovascular causes. The secondary outcomes consisted of the individual components of the primary outcome and all-cause death. Intensive blood pressure (BP) control significantly reduced the incidence of primary outcome event in patients with 10% ≤ ASCVD < 15% (hazard ratio (HR) 0.593; 95% confidence interval (CI) 0.361–0.975; *P* = 0.039) and ASCVD ≥ 15% (HR 0.778; CI 0.644–0.940; *P* = 0.009). Intensive BP control was also beneficial for the primary prevention of cardiovascular events in patients with an ASCVD risk of 7.5–10% (HR 0.187; 95% CI 0.040–0.862; *P* = 0.032). However, intensive treatment was associated with higher incidence of hypotension and acute renal failure in participants with ASCVD ≥ 15%. In patients without diabetes mellitus and prior stroke who had a 10-year risk of cardiovascular events above 10% based on the ASCVD risk score, intensive BP control played an important role in the reduction of major cardiovascular events. Additionally, intensive treatment would be beneficial for primary prevention in patients with ASCVD ≥ 7.5% without previous history of any cardiovascular disorders. Trial registration: ClinicalTrials.gov number; the trial is registered with NCT01206062.

## 1. Introduction

Hypertension is a prevalent chronic disease, especially in the elderly population, that leads to stroke, end-stage renal disease (ESRD), myocardial infarction (MI), congestive heart failure (CHF), and peripheral vascular disease [1].

Adequate control of hypertension plays a crucial role in cardiovascular disease (CVD) rate and subsequent mortality reduction and is much more cost-effective than treating cardiovascular events that result from uncontrolled hypertension [2]. Systolic blood pressure (SBP) is a more important predictor of cardiovascular events compared with diastolic blood pressure (DBP) [3]. It has been shown that antihypertensive treatment for an SBP of 140 mmHg or higher is associated with a reduced risk of death and CVD, and treatment is recommended for these patients [4]. However, some studies have suggested that intensive blood pressure (BP) reduction to a target SBP ≤ 120 mm Hg should be considered to decrease the risk of cardiovascular events in some special people [5, 6].

The Systolic Blood Pressure Intervention Trial [5] was a multicenter trial of 9361 adults ≥50 years of age, with a systolic blood pressures of ≥130 mm Hg and at least one additional cardiovascular risk factor, who were randomly assigned to either intensive (SBP target: ≤120 mm Hg) or standard (SBP target: ≤140 mm Hg) treatment group [7]. It was concluded that, in the patients with high CVD risk, targeting an SBP less than 120 mm Hg as compared with an SBP less than 140 mm Hg resulted in lower rates of fatal and nonfatal major cardiovascular events and death from any cause [5].

Clinical practice guidelines for hypertension treatment relied primarily on the BP levels. However, several studies have provided support for the positive role of CVD risk assessment in guiding BP-lowering treatment decisions [8, 9]. Several risk prediction tools have been developed to identify the patients at high risk of CVD, such as the Framingham Risk Score (FRS) and the Atherosclerotic Cardiovascular Disease (ASCVD) risk score. The ASCVD risk score is a formula developed by the American College of Cardiology and the American Heart Association for evaluation of the risk of future cardiovascular events [10].

In this study, we aimed to conduct a secondary analysis of SPRINT data in order to compare the effects of intensive BP control with an SBP target of less than 120 mmHg and standard BP control with an SBP target of less than 140 mmHg on cardiovascular outcomes in the patients who had different ASCVD risk scores at baseline.

## 2. Methods

### 2.1. Study Design and Population

This study was a post hoc analysis of SPRINT. The SPRINT data were obtained from the National Heart, Lung, and Blood Institute (NHLBI), Biologic Specimen and Data Repository Information Coordinating Center.

SPRINT was a randomized, controlled trial that was conducted at 102 clinical sites. In this study, a total of 9361 participants were enrolled. The patients were randomized into the intensive-treatment group with a target SBP of less than 120 mmHg and the standard-treatment group targeting an SBP of less than 140 mmHg (Figure 1) [5].

To be eligible for participation in the study, the patients were required to meet all the following criteria: (1) age ≥50 years; (2) an SBP of 130–180 mm Hg; and (3) an increased risk of cardiovascular events, which was defined by one or more of the following criteria: clinical or subclinical CVD other than stroke; chronic kidney disease (CKD), excluding polycystic kidney disease, with an estimated glomerular filtration rate (eGFR) of 20 to less than 60 ml/min/1.73 m^2^; a 10-year risk of CVD ≥ 15% on the basis of FRS; or age ≥ 75 years. The main exclusion criteria were one-minute standing SBP <110 mm Hg, proteinuria ≥1 g/day, diabetes mellitus (DM), history of stroke, polycystic kidney disease, eGFR < 20 ml/min/1.73 m^2^ or end-stage renal disease (ESRD), symptomatic heart failure (HF) within the past 6 months, and pregnancy [5].

The ASCVD risk score is a continuous score, ranging from 0% to 100%, to estimate the risk of cardiovascular events in the next 10 years on the basis of variables, including SBP, total cholesterol (TC), high-density lipoprotein cholesterol (HDL-C), age, sex, race, diabetes, and smoking status [11]. According to the ASCVD risk score, we divided the participants of SPRINT into four groups: ASCVD < 7.5%, 7.5% ≤ ASCVD < 10%, 10% ≤ ASCVD < 15%, and ASCVD ≥ 15%. This study has been approved by the national ethical committee by an approval number of IR.SUMS.MED.REC.1398.377 and conforms to the Declaration of Helsinki. All participants signed the consent form.

### 2.2. Intervention and Measurements

Participants were randomly assigned to an SBP target of either <140 mm Hg (the standard-treatment group) or <120 mm Hg (the intensive-treatment group). All major classes of antihypertensive drugs were included in the formulary. For participants in the intensive-treatment group, medications were adjusted to target an SBP <120 mm Hg. Medications for participants in the standard-treatment group were adjusted to target an SBP of 135–139 mm Hg, and the dose decreased if SBP was <130 mm Hg on a single visit or <135 mm Hg on two consecutive visits [5].

The mean of three BP measurements at an office visit while the patient was seated and after five minutes of quiet rest was considered as a basis for dose adjustment of drugs. Blood pressure measurements were done by an automated measurement system (Model 907, Omron Healthcare) [5].

Demographic data were obtained from participants at baseline. Clinical and laboratory data were recorded at baseline and then every 3 months. In addition, a structured interview was done every 3 months to obtain self-reported CVD outcomes [5].

### 2.3. Clinical Outcomes

The primary end point was a composite of nonfatal MI, acute coronary syndrome (ACS) not resulting in MI, stroke, acute decompensated HF, or death from cardiovascular causes [12]. The secondary outcomes were the individual components of the primary outcome and all-cause death [13].

### 2.4. Serious Adverse Events

Serious adverse events (SAEs) were defined as events that met any of the following criteria: (1) being fatal or life-threatening; (2) resulting in significant or persistent disability; (3) requiring or prolonged hospitalization; or (4) suffering important medical event that is judged to represent significant hazards to participants and may require medical or surgical intervention. Adverse events consisted of syncope, bradycardia, hypotension, electrolyte disturbances, and acute renal failure (AKI) which were evaluated at the emergency department [14].

### 2.5. Statistical Analysis

Statistical analysis was performed using the chi-square test, the one-way ANOVA test, and the proportional hazard cox regression model. A *P* value less than 0.05 was considered significant. SPSS version 22 (IBM SPSS, Armonk, NY, USA) was used to perform data analysis.

## 3. Results

### 3.1. Study Participants

We used data of 9361 patients who participated in the SPRINT trial. There were 869, 781, 1889, and 5822 patients with ASCVD < 7.5%, 7.5% ≤ ASCVD < 10%, 10% ≤ ASCVD < 15%, and ASCVD ≥ 15%, respectively. The participants with ASCVD ≥ 15% were older and had higher SBP, triglycerides (TG), and glucose levels. Regarding various parameters, no statistically significant differences were found between the intensive- and standard-treatment group in each ASCVD category. The demographic and clinical data of the cases are summarized in Table 1.

### 3.2. Clinical Outcomes

A primary outcome event was reported in 22 patients with ASCVD < 7.5%–12 in the standard-treatment group and 10 in the intensive-treatment group (hazard ratio (HR) with intensive treatment 0.668; 95% confidence interval (CI) 0.272–1.637; *P* = 0.378); 29 patients with 7.5% ≤ ASCVD < 10%–16 in the standard-treatment group and 13 in the intensive-treatment group (HR 0.659; 95% CI 0.294–1.478; *P* = 0.311); 71 patients with 10% ≤ ASCVD < 15%–45 in the standard-treatment group and 26 in the intensive-treatment group (HR 0.593; 95% CI 0.361–0.975; *P* = 0.039); and 440 patients with ASCVD ≥ 15%–246 in the standard-treatment group and 194 in the intensive-treatment group (HR 0.778; 95% CI 0.644–0.940; *P* = 0.009). Generally, intensive BP control had a significant role in the reduction of the primary outcome in the patients with ASCVD ≥ 10 (Table 2, Figure 2). Intensive BP control also reduced the incidence of HF (HR 0.61; 95% CI 0.44–0.84; *P* = 0.003) and CVD (HR 0.56; 95% CI 0.37–0.84; *P* = 0.006) in the total population regardless of ASCVD risk scores. The details of secondary outcomes are shown in Table 3. Additionally, in terms of primary prevention (those without previous cardiovascular disease), intensive treatment was beneficial in participants with ASCVD ≥ 7 5% (HR 0.187; 95% CI 0.040–0.862; *P* = 0.032).

### 3.3. Serious Adverse Events

SAEs consisted of hypotension, syncope, bradycardia, AKI, and electrolyte abnormality. Intensive treatment-related SAEs showed an increased risk of hypotension and syncope among the participants with ASCVD ≥ 15% and 10% ≤ ASCVD < 15%, respectively. The incidence of AKI was significantly higher in the patients with 7.5% ≤ ASCVD < 10% and ASCVD ≥ 15%. Additionally, in the total population, the risk of hypotension, AKI, and electrolyte abnormality significantly increased. ASCVD-stratified subgroup analysis of SAEs between intensive- and standard-treatment group is detailed in Table 4.

### 3.4. Patients at High ASCVD Risk

We did perform an analysis in the subpopulation of patients with an ASCVD risk ≥15 since they represent 62% of the total study population. Among them, 440 patients, 246 in the standard-treatment group and 194 in the intensive-treatment group (HR 0.778; 95% CI 0.644–0.940; *P* = 0.009), developed with a primary outcome. In addition, we performed a retrospective comparison of baseline characteristics between patients who had developed AKI and those who did not in the whole study population; those who had developed AKI had a lower eGFR (56.28% vs. 72.50%, *P* < .001) and a higher serum creatinine level (1.43 vs. 1.05, *P* < .001) compared to those who did not develop AKI. In fact, the presence of CKD increased the chance of AKI by 215%, and an eGFR below 62.04% predicted the occurrence of AKI with 66.77% sensitivity and 69.39% specificity (area under the curve, 0.715; *P* < .001, Figure 3).

## 4. Discussion

This study was a post hoc analysis of SPRINT, which investigated the effects of intensive BP treatment on clinical outcomes in patients with different baseline ASCVD risk scores. The results of this study suggested that the intensive control of SBP was able to decrease cardiovascular events in patients with ASCVD risk score of 10% and above. Furthermore, our study suggested that intensive treatment would be beneficial for primary prevention in patients with ASCVD ≥ 7.5%.

There is still debate as to whether the BP-lowering strategy should be determined on the basis of BP alone. Ogden et al. demonstrated that the absolute benefits of antihypertensive therapy depended not only on the BP level but also on the presence or absence of additional CVD risk factors [15]. The Cardiovascular Health Awareness Program in Canada also reported that management via stratification of risk factors for hypertensive patients reduced CVD mortality in comparison to the usual care [16]. However, many guidelines have not provided recommendations regarding risk-based strategies for hypertension management. This might be due to the lack of enough evidence in this regard. In addition, further studies are needed to determine a proper target of SBP in patients with hypertension who have various comorbidities and CVD risk at baseline [8, 17, 18].

Zhang et al. compared the effects of intensive BP control and standard treatment among the patients with different baseline Framingham Risk Score (FRS). Their study showed that, in high-risk participants, intensive BP treatment was effective in the risk reduction of the primary outcome. Furthermore, they concluded that the intensive treatment of BP was advantageous in the total population irrespective of the levels of FRS [13]. Although we used a different risk assessment system, our results also showed that the patients with a higher risk of CVD would benefit from intensive BP treatment.

Williamson et al. evaluated the effects of intensive treatment (SBP target <120 mmHg) versus standard treatment (SBP target <140 mmHg) in patients aged 75 years or older with hypertension, but without diabetes. They found that treating to an SBP target of less than 120 mmHg compared with an SBP target of less than 140 mmHg resulted in significantly lower rates of fatal and nonfatal major cardiovascular events and death from any cause [19]. In agreement with this observation, our analysis suggested that intensive BP control lessened the risk of CVD outcomes in the patients with higher ASCVD risk scores who were older.

In contrast to our study, the ACCORD trial did not identify an SBP target <120 mmHg advantageous for patients with type 2 DM, with the exception of decreased stroke risk [20]. However, in Sprint's study, the patients with DM were excluded.

Attar et al. observed that intensive treatment led to a significant reduction in the primary outcome events in patients with FRS ≥ 10% [8]. Our results are consistent with this study, as we found that intensive BP control could positively affect the hypertensive patients with ASCVD ≥ 10%.

Although intensive BP treatment can avert cardiovascular events, it can cause some serious adverse health consequences [21–24]. In SPRINT's study, it was shown that the rates of eGFR reduction ≥30% and below 60 ml/min/1.73 m^2^ and the incidence of SAEs, such as hypotension, syncope, AKI, and electrolyte abnormalities in patients without CKD at baseline were more common in the intensive therapy group [25]. Our study indicated that the incidence of hypotension and AKI was higher among the patients with ASCVD ≥ 15%, which highlighted the fact that the intensive treatment of BP could lead to an increased risk of SAEs.

Similarly, in Accord's study, patients with an achieved SBP target of about 120 mmHg had an increased risk of SAEs compared to the patients remaining at an on-treatment SBP of about 133 mmHg [20]. Zhang et al. reported that the risk of SAEs associated with BP treatment significantly increased among the total population, intermediate-risk patients, and high-risk participants [13].

The limitation of our study was that the participants aged under 50 years and the patients with a positive history of stroke, ESRD, diabetes, and congestive HF were excluded. Therefore, the findings of this study could not be generalized to these patients.

## 5. Conclusions

In conclusion, our study showed that, in the patients aged under 75 years without DM, ESRD, or prior stroke who had a 10-year risk of cardiovascular events above 10% on the basis of the ASCVD risk score, intensive BP control with an SBP target of less than 120 mmHg significantly reduced the incidence of major cardiovascular events. However, it might be accompanied with an increased risk of SAEs such as hypotension and AKI. It has also been shown that intensive treatment would be beneficial for primary prevention in patients with ASCVD ≥ 7.5%. Totally, our findings suggested that an antihypertensive treatment strategy on the basis of a combination of CVD risk assessment and BP level could bring benefits to the patients.

## Figures and Tables

**Figure 1:** CONSORT flow diagram.

**Figure 2:** ASCVD-stratified Kaplan–Meier curve analysis was performed to compare the primary outcome between the intensive-treatment group and the standard-treatment group among the patients with ASCVD < 7.5%, 7.5% ≤ ASCVD < 10%, 10% ≤ ASCVD < 15%, and ASCVD ≥ 15%. (a) Hazard function for patterns 1-2 ASCVD groups: ASCVD < 7.5. (b) Hazard function for patterns 1-2 ASCVD groups: 7.5 ≤ ASCVD <10. (c) Hazard function for patterns 1-2 ASCVD groups: 10 ≤ ASCVD < 15. (d) Hazard function for patterns 1-2 ASCVD groups: ASCVD ≥ 15.

**Figure 3:** ROC curve for prediction of kidney injury based on eGFR is demonstrated. An eGFR below 62% could be defined as a cut-off point for predicting AKI development with intensive blood pressure reduction.

**Table 1:** Demographic and clinical characteristics of participants with different baseline ASCVD risk scores.

Characteristics	ASCVD below 7.5%		ASCVD equal to or greater than 7.5% and less than 10%		ASCVD equal to or greater than 10% and less than 15%		ASCVD equal to or greater than 15%.	
	Intensive	Standard	Intensive	Standard	Intensive	Standard	Intensive	Standard
N	438 (9.4)	431 (9.2)	396 (8.5)	385 (8.2)	936 (20.0)	953 (20.4)	2908 (62.2)	2914 (62.2)
ASCVD%	5.44 ± 1.43	5.41 ± 1.53	8.84 ± 0.73	8.73 ± 0.73	12.49 ± 1.45	12.48 ± 1.41	30.16 ± 13.75	30.07 ± 13.59
Age, y	57.35 ± 4.24	57.07 ± 4.42	60.26 ± 4.80	59.81 ± 5.02	62.25 ± 5.68	62.35 ± 5.75	72.39 ± 8.35	72.40 ± 8.40
Female	298 (17.7)	288 (17.5)	207 (12.3)	194 (11.8)	345 (20.5)	337 (20.4)	834 (49.5)	829 (50.3)

Smoking status								
Never	237 (13.3)	252 (12.2)	230 (9.9)	199 (9.6)	435 (21.2)	443 (21.4)	1139 (55.6)	1178 (56.9)
Former	134 (6.8)	149 (7.5)	154 (7.8)	148 (7.4)	377 (19.1)	397 (19.9)	1312 (66.4)	1302 (65.2)
Current	31 (4.9)	30 (5.0)	39 (6.1)	38 (6.3)	123 (19.2)	112 (18.6)	867 (69.9)	446 (69.8)
SBP, mmHg	131.1 ± 14.5	129.9 ± 14.1	133.3 ± 13.6	133.6 ± 13.3	136.5 ± 14.7	136.7 ± 13.9	142.8 ± 15.5	142.8 ± 15.2
DBP, mmHg	80.6 ± 10.7	80.0 ± 10.9	80.2 ± 11.0	80.3 ± 10.3	80.5 ± 11.0	80.5 ± 11.3	76.8 ± 12.2	78.0 ± 12.3
BMI, kg/m^2^	31.9 ± 6.7	31.9 ± 6.4	31.5 ± 6.2	31.4 ± 6.8	30.9 ± 6.2	30.9 ± 5.7	29.0 ± 5.2	28.8 ± 5.2
TC, mg/dL	195.5 ± 42.7	194.7 ± 44.3	194.7 ± 41.1	192.8 ± 37.7	191.8 ± 40.7	190.4 ± 40.3	188.2 ± 41.3	188.8 ± 40.9
HDL, mg/dL	54.7 ± 15.3	55.0 ± 14.9	53.2 ± 15.1	53.2 ± 14.4	52.1 ± 12.9	51.9 ± 14.0	52.9 ± 14.4	52.7 ± 14.7
TG, mg/dL	123.8 ± 64.9	125.9 ± 79.4	124.4 ± 66.0	119.4 ± 67.6	124.0 ± 102.0	127.9 ± 87.5	125.2 ± 85.1	128.0 ± 102.2
Glucose, mg/dL	96.9 ± 10.8	97.4 ± 10.6	98.3 ± 11.7	96.7 ± 11.4	97.8 ± 12.6	98.2 ± 11.6	99.5 ± 14.6	99.4 ± 14.4
ALCR, mg/g	24.9 ± 84.1	35.1 ± 140.9	24.5 ± 75.6	32.3 ± 148.3	35.8 ± 177.9	39.3 ± 183.2	52.2 ± 197.7	43.7 ± 144.0
EGFR	75.6 ± 20.5	75.1 ± 21.6	75.3 ± 22.0	77.4 ± 21.0	76.6 ± 20.9	74.8 ± 19.7	69.0 ± 19.9	69.4 ± 20.1
CKD history	90 (6.8)	96 (7.3)	91 (6.8)	71 (5.4)	185 (13.9)	198 (15.0)	968 (72.5)	951 (72.3)
CVD history	80 (8.5)	79 (5.4)	64 (6.8)	63 (6.7)	140 (14.9)	175 (18.7)	656 (69.8)	620 (66.2)

N_AGENTS								
0	68 (15.7)	46 (10.0)	53 (12.3)	52 (11.6)	111 (25.7)	121 (26.9)	200 (46.3)	232 (51.6)
1	136 (10.0)	124 (8.9)	118 (8.6)	113 (8.1)	254 (18.6)	263 (18.9)	857 (62.8)	888 (64.0)
2	131 (7.9)	168 (10.3)	140 (8.4)	127 (7.8)	322 (19.3)	307 (18.9)	1072 (64.4)	1025 (63.0)
3	79 (8.3)T	77 (8.0)	70 (7.3)	74 (7.7)	195 (20.4)	196 (20.3)	612 (64.0)	617 (64.0)
4	23 (9.1)	17 (7.0)	15 (5.9)	17 (7.0)	54 (21.3)	65 (26.6)	161 (63.6)	154 (59.4)
5	1 (16.7)	0	0	2 (20)	0	1 (10)	5 (83.3)	7 (70.0)
6	0	0	0	0	0	0	1 (100)	0
Statin	153 (7.7)	167 (8.0)	147 (7.4)	134 (6.5)	357 (18.0)	400 (19.3)	1321 (66.8)	1375 (66.2)

Data were presented as mean ± SD or number (%) for continuous and categorical variables, respectively. ASCVD: Atherosclerotic Cardiovascular Disease, SBP: systolic blood pressure, DBP: diastolic blood pressure, BMI: body mass index, TC: total cholesterol, HDL: high density lipoprotein, TG: triglycerides, ALCR: albumin-to-creatinine ratio, EGFR: estimated glomerular filtration rate, CKD: chronic kidney disease, CVD: cardiovascular disease, N_AGENTS: number of antihypertensive agents.

**Table 2:** Primary outcome in the intensive- and standard-treatment group.

Subgroups	Primary outcome		
ASCVD < 7.5%	Number		
Standard	Yes	12	Reference
	No	419	
Intensive	Yes	10	0.668 (0.272–1.637), 0.378
	No	428	

7.5% ≤ ASCVD < 10%			
Standard	Yes	16	Reference
	No	369	
Intensive	Yes	13	0.659 (0.294–1.478), 0.311
	No	383	

10% ≤ ASCVD < 15%			
Standard	Yes	45	Reference
	No	908	
Intensive	Yes	26	0.593 (0.361–0.975), **0.039**
	No	910	

ASCVD ≥ 15%			
Standard	Yes	246	Reference
	No	2668	
Intensive	Yes	194	0.778 (0.644–0.940), **0.009**
	No	2714	

Data were presented as hazard ratio (95% confidence interval), *P* value. The bold *P* value data indicates its significance. ASCVD: Atherosclerotic Cardiovascular Disease.

**Table 3:** Secondary outcomes in the intensive- and standard-treatment group.

Group	ASCVD%	Secondary outcomes				
		MI	Non-MI ACS	Stroke	HF	CVD death
Intensive/standard	<7.5%	0.39 (0.07–2.01), 0.261	0.01 (0.00–1295), 0.469	3.84 (0.42–34.36), 0.229	0.95 (0.23–3.82), 0.949	0.96 (0.13–6.81), 0.967
	7.5%–10%	0.95 (0.27–3.30), 0.945	1.45 (0.24–8.10), 0.681	0.24 (0.02–2.14), 0.202	1.87 (0.17–20.68), 0.608	0.47 (0.11–1.90), 0.296
	10%–15%	0.48 (0.20–1.11), 0.087	0.58 (0.17–1.98), 0.386	1.79 (0.52–6.12), 0.341	0.51 (0.21–1.19), 0.123	0.53 (0.14–1.47), 0.188
	≥15%	0.92 (0.68–1.24), 0.585	1.13 (0.69–1.87), 0.611	0.81 (0.56–1.18), 0.292	0.60 (0.42–0.86), **0.006**	0.58 (0.36–0.93), **0.024**
	Total	0.83 (0.63–1.09), 0.183	0.99 (0.64–0.154), 0.994	0.88 (0.62–1.24),0.472	0.61 (0.44–0.84), **0.003**	0.56 (0.37–0.84), **0.006**

Data were presented as hazard ratio (95% confidence interval), *P* value. The bold *P* value data indicates its significance. ASCVD: Atherosclerotic Cardiovascular Disease, MI: myocardial infarction, ACS: acute coronary syndrome, HF: heart failure, CVD: cardiovascular disease.

**Table 4:** Serious adverse events in the intensive- and standard-treatment group.

ASCVD	Hypotension	Syncope	Bradycardia	Acute renal failure	Electrolyte abnormality
< 7.5%					
Standard	Reference				
Intensive	2.88 (0.58–14.29), 0.194	0.95 (0.23–3.82), 0.950	0.47 (0.04–5.20), 0.540	0.83 (0.30–2.31), 0.734	2.45 (0.95–6.32), 0.063

7.5%–10%					
Standard	Reference				
Intensive	2.55 (0.67–9.63), 0.166	2.33 (0.45–12.14), 0.306	0.89 (0.12–6.36), 0.908	4.92 (1.07–22.46), **0.040**	1.59 (0.75–3.38), 0.222

10%–15%					
Standard	Reference				
Intensive	1.02 (0.46–2.28), 0.945	3.27 (1.30–8.20), **0.011**	1.95 (0.87–4.38), 0.104	1.61 (0.86–3.01), 0.137	1.37 (0.75–2.52), 0.310
≥15%					
Standard	Reference				
Intensive	1.17 (01.20–2.44), 0.003	1.16 (0.84–1.60), 0.364	1.11 (0.78–1.57), 0.548	1.67 (1.28–2.16), <**0.001**	1.28 (0.97–1.68), 0.071

Total population					
Standard	Reference				
Intensive	1.66 (1.22–2.26), **0.001**	1.33 (0.99–1.78), 0.051	1.18 (0.87–1.62), 0.279	1.65 (1.31–2.08), <**0.001**	1.37 (1.09–1.72), **0.006**

Data were presented as hazard ratio (95% confidence interval), *P* value. The bold *P* value data indicates its significance. ASCVD: Atherosclerotic Cardiovascular Disease.

## Data Availability

The SPRINT data were obtained from the National Heart, Lung, and Blood Institute (NHLBI) Data Repository (https://biolincc.nhlbi.nih.gov/studies/sprint/).

## Abbreviations

CVD: Cardiovascular disease
SBP: Systolic blood pressure
SPRINT: Systolic Blood Pressure Intervention Trial
ASCVD: Atherosclerotic Cardiovascular Disease
MI: Myocardial infarction
ACS: Acute coronary syndrome
HF: Heart failure
BP: Blood pressure
HR: Hazard ratio
CI: Confidence interval
ESRD: End-stage renal disease
CHF: Congestive heart failure
DBP: Diastolic blood pressure
FRS: Framingham Risk Score
NHLBI: National Heart, Lung, and Blood Institute
CKD: Chronic kidney disease
EGFR: Estimated glomerular filtration rate
DM: Diabetes mellitus
TC: Total cholesterol
HDL-C: High density lipoprotein cholesterol
SADE: Serious adverse events
AKI: Acute renal failure
TG: Triglycerides.
